The article "Analysis of DNA Sequence Classification Using CNN and Hybrid Models" was published in 2021. Journal: Comput Math Methods Med.

# Analysis of DNA Sequence Classification Using CNN and Hybrid Models

**DOI:** 10.1155/2021/1835056

**Published:** 2021-07-15

**Authors:** Hemalatha Gunasekaran, K. Ramalakshmi, A. Rex Macedo Arokiaraj, S. Deepa Kanmani, Chandran Venkatesan, C. Suresh Gnana Dhas

**Affiliations:** ^1^IT Department, University of Technology and Applied Sciences, Oman; ^2^Department of Computer Science and Engineering, Alliance School of Engineering and Design, Alliance University, Bangalore, Karnataka, India; ^3^Department of Information Technology, Sri Krishna College of Engineering and Technology, Coimbatore, Tamil Nadu, India; ^4^Department of Electronics and Communication Engineering, KPR Institute of Engineering and Technology, Coimbatore, Tamil Nadu, India; ^5^Department of Computer Science, Ambo University, Ambo, Post Box No.: 19, Ethiopia

## Abstract

In a general computational context for biomedical data analysis, DNA sequence classification is a crucial challenge. Several machine learning techniques have used to complete this task in recent years successfully. Identification and classification of viruses are essential to avoid an outbreak like COVID-19. Regardless, the feature selection process remains the most challenging aspect of the issue. The most commonly used representations worsen the case of high dimensionality, and sequences lack explicit features. It also helps in detecting the effect of viruses and drug design. In recent days, deep learning (DL) models can automatically extract the features from the input. In this work, we employed CNN, CNN-LSTM, and CNN-Bidirectional LSTM architectures using Label and *K*-mer encoding for DNA sequence classification. The models are evaluated on different classification metrics. From the experimental results, the CNN and CNN-Bidirectional LSTM with *K*-mer encoding offers high accuracy with 93.16% and 93.13%, respectively, on testing data.

## 1. Introduction

The world has 1.6 million viruses and viruses like HIV, Ebola, SARS, MERS, and COVID-19 that jumps from mammals and humans. The author provides a detailed study about the influence of COVID-19 in numerous sectors [1]. Due to the effect of globalisation and intense mobilisation of the global population, it is likely that new viruses can emerge and can spread across as fast as the current COVID-19. Identifying the pathogens earlier will help prevent an outbreak like COVID-19 and assist in drug design [2]. Therefore, DNA sequence classification plays a vital role in computational biology. When a patient is infected by the virus, the samples collected from the patient and the genomes are sequenced. The sequenced genomes will be compared in the GenBank (NCBI) to identify the pathogens. The GenBank maintains a BLAST server to check the similarity of the genome sequence. It has 106 billion nucleoid bases from 108 million different sequences, with 11 million new ones added last year [3]. Suppose the DNA sequences increase exponentially, machine learning techniques are used for DNA sequence classification. Any living organism's blueprint is DNA (deoxyribonucleic acid).

The article "Analysis of DNA Sequence Classification Using CNN and Hybrid Models" was published in 2021. Journal: Comput Math Methods Med.

Adenine (A), cytosine (C), guanine (G), and thymine (T) are the four nucleotides that makeup DNA (T). These are called the building blocks of DNA. The DNA of each virus is unique, and the pattern of arrangement of the nucleotides determines the unique characteristics of a virus [4]. DNA appears as single-stranded or double-stranded (as shown in Figure 1). Each form of nucleotide binds to its complementary pair on the opposite strand in double-stranded DNA. Adenine and thymine form a pair, while cytosine and guanine form a pair. Ribonucleic acid (RNA) may be single-stranded or double-stranded. In RNA, uracil (U) replaces the thymine (T). Therefore, the genome is the sequence of nucleotides (A, C, G, T) for DNA virus and (A, C, U, G) for RNA virus [5].

The DNA sequence is very long, having a length of around 32,000 nucleotides maximum, and it is challenging to understand and interpret. This raw DNA sequence cannot give as input to the CNN for feature extraction. It has to be converted into numerical representation before it is processed in the CNN. The encoding method also plays a vital role in classification accuracy. Two encoding methods used in this paper: to begin, label encoding, in which each nucleoid in a DNA sequence is identified by a unique index value, preserving the sequence's positional information [6]. Secondly, *K*-mers are generated for the DNA sequence, and the DNA sequence is converted into English-like statements. Thus, any text classification technique can be used for DNA classification. Feature engineering is fundamental for any model to produce good accuracy. In the machine learning models, feature extraction is done manually [7]. But as the complexity of the data increases, the manual feature selection may lead to many problems like selecting features that do not lead to the best solution or missing out on essential features. Automatic feature selection can be used to overcome this issue. CNN [8] is one of the best deep-learning techniques used to extract key features from the raw dataset.

Most importantly, from the DNA dataset, the key features are not very clear. The extracted features from the raw DNA sequence are fed into the LSTM and bidirectional LSTM models for classification. This paper compared the accuracy and the other metrics of the CNN model with hybrid models such as CNN-LSTM [9] and CNN-Bidirectional LSTM [10]. The same models are run with both label encoding and *K*-mer encoding to conclude which encoding is best for the DNA sequence.

The article "Analysis of DNA Sequence Classification Using CNN and Hybrid Models" was published in 2021. Journal: Comput Math Methods Med.

The author proposed deep learning methods like CNN, DNN, and N-gram probabilistic model to classify DNA sequence. A new approach to extract the features using the random DNA sequence based on the distance measure is proposed. Finally, they evaluated the model with four different datasets, namely, COVID-19, AIDS, influenza, and hepatitis C [11]. This study presented the classification of mutated DNA sequence to identify the origin of viruses using the extreme gradient boosting algorithm. They achieved an accuracy of 89.51% using a hybrid approach of XGBoost learning to classify DNA sequence [12]. The N4-methylcytosine from the DNA sequence is predicted using the deep learning model's feature selection and stacking method and the area under the curve greater than 0.9 [13]. The author proposed a classification model for DNA barcode fragment and short DNA sequence. The author created a free Python package to perform alignment-free DNA sequence classification. The developed model used the *K*-mer feature extraction method and optimal machine learning model for type and achieved an accuracy of around 99% [14]. The linear classifier like Multinomial Bayes, Markov, Logistic Regression, and Linear SVM is used to classify the partial and complete genomic sequence of the HCV dataset is proposed. The author evaluated and compared the results for different *K*-mer size [15]. In [16], the author presented the method for predicting SARS-CoV-2 using the deep learning architecture with 100% specificity. The author proposed a new algorithm for improving code construction that is distinct from the DNA sequence obtained. They replaced brute force decoding with syndrome decoding [17]. In this study, the author used an ensemble decision tree approach to classify the complex DNA sequence dataset. The author used the XGBoost and Random Forest ensemble techniques to obtain a 96.24% and 95.11% accuracy, respectively [18]. In this work, machine learning methods are used to classify the DNA sequence of cancer patients, and the Random Forest algorithm performs better [19]. The author proposed a CNN-based model to classify exons and introns in the human genomes and achieved a testing rate of 90% [20]. The author used CNN for metagenomics gene prediction. The author trained 10 CNN model on 10 datasets.

The ORFs (noncoding open reading frames) were extracted from each fragment and converted into numerical to give input to the CNN model. GC content of the fragment is used as the feature matrix. The author achieved an accuracy of around 91% on the testing data [21]. They used deep learning to classify genetic markers for liver cancer from the hepatitis B virus DNA sequence in this analysis, and the training dataset had an accuracy of about 96.83% [22]. The DL architecture is proposed to classify three genome types of the coding region, long noncoding region, and pseudoregions and achieve an average accuracy of 84% [23]. The author used the one-hot encoding technique to represent the sequences of DNA. The model is evaluated with 12 DNA sequence dataset which contains binary classification [24]. In [25], the author proposed the DL architecture to predict the short sequences in 16s ribosomal DNA and achieves the maximum accuracy of 81.1%. The spectral sequence representation-based deep learning neural network was proposed [26]. The author tested the model on a dataset of 3000 16S denes and compared the results with GRAN (General Regression Neural Network). The author found the best hyperparameters for the model, which obtained better results. The role of big data plays a vital role in intelligent learning [27]. From the literature review, the research gap is identified that for classification of different DNA sequencing for other diseases, using the generalised model is not carried out. By considering the fact, the main contribution of this study can be summarised as follows:

1. To the best of our knowledge, this is the first time a deep learning model was developed to classify COVID, MERS, SARS, dengue, hepatitis and influenza
2. To represent sequences, we used both Label and *K*-mer encoding, which preserve the position information of each nucleotide in the sequence
3. Three different deep learning architectures for classifying DNA sequences are presented in this paper: CNN, CNN-LSTM, and CNN-Bidirectional LSTM

Section 2 delves into the proposed deep learning algorithm and dataset acquisition and data preprocessing to show how nucleotide sequences are interpreted as input to the model—the findings of the model and validation studies presented in Section 3.  Section 4 contains some observations and discussion.

The article "Analysis of DNA Sequence Classification Using CNN and Hybrid Models" was published in 2021. Journal: Comput Math Methods Med.

## 2. Methodology

### 2.1. Data Collection

The complete DNA/Genomic sequence of the viruses like COVID, SARS, MERS, dengue, hepatitis, and influenza obtained from the public nucleotide sequence database: “The National Centre for Biotechnology Information (NCBI)” (https://www.ncbi.nlm.nih.gov). The format of the DNA sequence data is FASTA file, and the metadata is provided in Table 1. The length of the sequence ranges from 8 to 37,971 nucleoids. The class distribution of each class with the number of samples is shown in Figure 2. The sample DNA sequences from the dataset with the complete genomic sequence of a virus, the length of the sequence, and the class labels are shown in Figure 3.

From the dataset, it is clearly showing that there is an imbalanced dataset problem. SMOTE (Synthetic Minority Oversampling Technique) is employed [28] to handle this problem. In our dataset, MERS and dengue DNA sequences are deficient in numbers. Synthetic samples for the minority classes like MERS and dengue are generated using the SMOTE algorithm to match the majority class closely. SMOTE picks a minority class instance randomly and searches for its *k* closest minority class neighbors. The synthetic instance is then constructed by randomly selecting one among the *k* nearest neighbors *b* and connecting *a* and *b* within the feature space to supply a line segment. The synthetic instances are created by combining the two chosen examples, *a* and *b*, in a convex way. This procedure can be used to make an artificial instance for the minority classes.

### 2.2. Data Preprocessing

Preprocessing data is the most critical step in most machine learning and deep learning algorithms that involve numerical rather than categorical data. The genomic sequence in the DNA dataset is categorical. There are many techniques available to convert the categorical data to numerical. The encoding technique is the process of converting the categorical data of nucleotide into numerical form. In this paper, label encoding and *K*-mer encoding are used to encode the DNA sequence. The effect of the encoding technique on the classification accuracy is analysed. In Label encoding, each nucleotide in the DNA sequence is assigned an index value like (A-1, C-2, G-3, and T-4) as shown in Figure 4. The entire DNA sequence is converted into an array of numbers using LabelBinarizer ().

In *K*-mer encoding technique, the raw DNA sequence is converted into an English-like statement by generating *K*-mers for the DNA sequence. Each DNA sequence is transformed into a *K*-mer of size *m*, as shown in Figure 5, and all the *K*-mers generated are concatenated to form a sentence [29]. Now, natural language processing technique can be used to classify the DNA sequence. The word embedding layer is used in this study to transform the *K*-mer sentence into a dense feature vector matrix.

### 2.3. Classification Models

In this work, three different classification models CNN, CNN-LSTM, and CNN-Bidirectional LSTM are used for DNA sequence classification.

The label encoding and *K*-mer techniques are used to encrypt the DNA sequence, which preserves the position information of each nucleotide in the sequence. The embedding layers is used to embed the data from the above two techniques. The CNN layer is used as the feature extraction stage, and it is given as the input for LSTM and bidirectional LSTM for classification. The workflow for the proposed work is shown in Figure 6.

The article "Analysis of DNA Sequence Classification Using CNN and Hybrid Models" was published in 2021. Journal: Comput Math Methods Med.

#### 2.3.1. CNN

CNN is a common deep-learning technique that can yield cutting-edge results for most classification problems [30, 31]. CNN performs well not only on image classification, but it can also produce good accuracy on text data. Mainly, CNN is used to automatically extract the features from the input dataset, in contrast to machine learning models, where the user needs to select the features 2D CNN [32], and 3D CNN is used for image and video data, respectively, whereas 1D CNN is used for text classification. The DNA sequence is treated as a sequence of letters (nucleoids A, C, G, and T). Since CNN can work only with numerical data, the DNA sequence is converted into numerical values by applying one hot encoding or label encoding. The CNN architecture uses a series of convolutional layers to extract features from the input dataset. Max pooling layer after each convolutional layer and the dimensions of extracted features are reduced. In the convolutional layer, the size of the kernel plays a significant role in function extraction. The model's hyperparameters are the number of filters and kernel size [33].  Table 2 shows the summary of the complete architecture of the proposed CNN model. The first layer is the embedded layer with dimension 8. This layer converts the words to a vector space model based on how often a word appears close to other words. The embedding layer uses random weights to learn embedding for all of the terms in the training dataset [34]. Two convolutional layers are added to the model with filters of 128 and 64, along with the kernel of size (2 × 2) with ReLU as an activation function for feature extraction. The feature map dimensions are reduced by adding a max pooling layer of size (2 × 2). Finally, the feature maps are converted into single-column vector using the flatten layer. The output is passed to a dense layer with neurons 128 and 64, respectively. The softmax function is used as the classification layer, which can perform well for the multiclass problem. The softmax layer consists of *N* units, where the *N* is the number of units. Each unit is fully connected with pervious layer and computes the probability of the each class on *N* by means of Equation (1).

(1) $$\begin{array}{c} \text{Softmax}=\frac{e^{w_{Nx}+b_{N}}}{\sum_{m=1}^{N}e^{w_{mx}+b_{m}}}. \end{array}$$

*W*_*m*_ is the weight matrix connecting the *m*^th^ unit to the previous layer, *x* is the last layer's output, and *b*_*m*_ is the *m*^th^ unit's bias.

The article "Analysis of DNA Sequence Classification Using CNN and Hybrid Models" was published in 2021. Journal: Comput Math Methods Med.

#### 2.3.2. CNN-LSTM

Long short-term memory (LSTM) is a recurrent neural network (RNN) that can learn long-term dependencies in a sequence and is used in sequence prediction and classification. It includes a series of memory blocks known as cells, each of which comprises three gates: input, output, and forget. The LSTM will selectively remember and forget things in this case [35].  Figure 7 depicts the LSTM model's overall architecture. It is capable of learning and recognises the long sequence. The current state is calculated using Equation (2),

(2) $$\begin{array}{c} h_{t}=f\left(h_{t-1},X_{t}\right), \end{array}$$

where *X*_*t* is the input state, *h*_*t* is the current state, and *h*_(*t* − 1) is the previous state.

In the LSTM, the forget gate is in charge of removing any information from the cell state. When detailed information becomes invalid for the sequence classification, the forget gate outputs a value of 0, indicating to remove the data from the memory cell. This gate takes two inputs, h_(t-1) (input from the previous state) and X_t (input from the current state). The input will be multiplied by a weight and added with bias. Finally, the sigmoid function is applied. The sigmoid function outputs the value ranging from 0 to 1. The input gate in the LSTM is responsible for adding all the relevant value to the cell state. It involves two activation functions: firstly, the sigmoid function controls what values add to the cell state. The second function is the tanh function, which returns values in the range of -1 to +1, indicating all possible values applied to the cell state. The output gate in LSTM decides what value can be in the output by employing the sigmoid activation function and tanh activation function to the cell state. The LSTM layer with 100 memory units is added after the convolutional layers to predict the classification labels in our model. The features extracted by the convolutional layer is given as an input to the LSTM layer for classification. In many NLP tasks, CNN and LSTM are combined into a hybrid model to improve the accuracy of the classification [36]. This hybrid model has produced surprising results in text classification. The LSTM model includes dropout layers and regularisation techniques to reduce the overfitting problem.

#### 2.3.3. CNN-Bidirectional LSTM

The bidirectional LSTM + CNN hybrid model is used for DNA sequence classification. The model uses CNN for feature extraction and bidirectional LSTM for classification. The bidirectional LSTM contains two RNN, one to learn the dependencies in the forward sequence and another to learn the dependencies in the backward sequence [37]. The architecture of the bidirectional LSTM is given in Figure 8.

The article "Analysis of DNA Sequence Classification Using CNN and Hybrid Models" was published in 2021. Journal: Comput Math Methods Med.

## 3. Results and Discussion

The proposed models are experimented with using the Tesla P100 GPU processor with a RAM size of 16280 MB. The dataset consists of 66,153 inputs divided into training, validation, and testing ratio of 70%, 10%, and 20%, respectively. The training set consists of 46307, and the validation set consists of 6615, and the testing set consists of 13231 samples. The maximum sequence length is 2000, and the vocabulary size is 8972. In the training phase, the binary crossentropy function is used as the loss function. This loss function calculates the error between the actual output and the target label, on which the training and update of the weights are done. We tested the CNN, CNN-LSTM, and CNN-bidirectional LSTM by varying the values of different hyperparameters like filters, filter size, the number of layers, and the embedding dimension. Grid search cross validation is the most widely used parameter optimisation method to select the best parameters for the model. The best parameters of all three models are the numbers of filters 128, 64, and 32 in each layer. The size of the filter is 2 × 2, training batch size of 100, training epochs of 10, embedding dimension of 32, and *K*-mer size of 6. The classification models are evaluated using different classification metrics like accuracy, precision, recall, F1 score, sensitivity, and specificity. The above-said metrics are calculated from the confusion matrix by obtaining True Positive_Gene_ (TP_Gene_), True Negative_Gene_ (TN_Gene_), False Positive_Gene_ (FP_Gene_), and False Negative_Gene_ (FN_Gene_). The confusion matrix for the proposed label encoding and *K*-mer encoding is shown in Figure 9.

Based on the above classification states, the formulas for the different metrics are given below:

(3) $$\begin{array}{c} \text{Accuracy}=\frac{\text{TPGene}+\text{TNGene}}{\text{TPGene}+\text{TNGene}+\text{FPGene}+\text{FNGene}},\\ \text{Specificity}=\frac{\text{TNGene}}{\text{TNGene}+\text{FPGene}},\\ \text{Sensitivity}=\frac{\text{TPGene}}{\text{TPGene}+\text{FNGene}},\\ \text{Precisio}=\frac{\text{TPGene}}{\text{TPGene}+\text{FPGene}}. \end{array}$$

Among the actual positive sequences, sensitivity is the proposition of a sequence defined as positive by the model. Because of the high sensitivity, a few positive cases are expected to be false negatives. The F1-score is the average of recall and precision. Precision is the percentage of documents positively identified as positive by the model. Specificity specifies how well the model determines the negative cases.  Figure 10 shows the accuracy of CNN and the hybrid models CNN-LSTM and CNN-Bidirectional LSTM. CNN offers higher accuracy only when the DNA sequences are encoded using label encoding. At the same time, LSTM and bidirectional LSTM provide more accuracy when DNA sequences are encoded using *K*-mer. We found that all the testing accuracies in the label encoding method are less than the training accuracy. In the case of *K*-mer encoding, the testing accuracy rates are more significant than the training accuracy. The results show that the use of the encoding method plays a vital role in classification accuracy.  Figure 11 shows that the accuracy of the CNN model increases for each epoch and continues to remain the same after epoch 10, whereas the accuracy of CNN-LSTM using *K*-mer encoding drops and increases at every epoch. It remains unstable throughout the training phase. The loss values for training and testing data for all three models, namely, CNN, CNN-LSTM, and CNN-Bidirectional LSTM with label encoding and *K*-mer encoding, are shown in Figure 12.

The article "Analysis of DNA Sequence Classification Using CNN and Hybrid Models" was published in 2021. Journal: Comput Math Methods Med.

### 3.1. Model Comparison and Analysis

The proposed method is compared with the different techniques to prove the robustness of the model: the proposed models, namely, CNN, CNN-LSTM, and CNN-Bidirectional LSTM. The CNN and CNN-bidirectional LSTM provide better accuracy of 93.16% and 93.13%, respectively. The achieved accuracy is obtained in classifying the six different classes. The models considered for the performance analysis from the literature are trained to classify up to three categories. The model [24] proposed by the authors is for classifying binary classification with an accuracy of 88.99%. In [12], the author has presented the model to classify five types of the chromosome by using the XGboost algorithm with an accuracy of 88.82%. In [11], the SARS-Cov2 cells are classified using the CNN, which obtained an accuracy of 88.82%. The comparative analysis is shown in Figure 13. The above experimental results clearly show that the proposed model works well for the DNA sequence classification. The 1D-CNN works well to classify DNA sequence classification to find the valuable pattern from the text data. It is found that the CNN model is extracting the features, which is very useful for the classification algorithm to classify the actual classes with an accuracy of 93.16%. The CNN bidirectional LSTM provides the next better accuracy with 93.13%, which has the advantages of holding the long-term dependencies compared to the CNN models by encoding sequence using the *K*-mer technique.

Further, the experiments carried out different class labels a, b, c, d, e, and f provided in Table 3. CNN with label encoding offers a better precision rate for the classification of class “a.” The CNN LSTM provides better precision than CNN and CNN-Bidirectional LSTM. This condition becomes inverse with *K*-mer encoding for other classes. We conclude that when the class samples are high, CNN with label encoding offers a high precision rate, and when the class samples are less, CNN with *K*-mer encoding provides a higher precision rate. The recall value for all the models with *K*-mer encoding is high irrespective of class labels. If a high recall rate is preferred for a classification model, then *K*-mer coding can be used. A higher sensitivity rate of 99.95% is obtained for class “a” with CNN–bidirectional LSTM model with label encoding. Thus, to obtain higher recall and sensitivity value for class with more sample, bidirectional LSTM with label encoding will be a good choice. CNN with label encoding offers a higher specificity rate for all the class irrespectively of class size.

The article "Analysis of DNA Sequence Classification Using CNN and Hybrid Models" was published in 2021. Journal: Comput Math Methods Med.

## 4. Conclusion

This paper compared three deep-learning methods, namely, CNN, CNN-LSTM, and CNN-bidirectional LSTM, with label encoding and *K*-mer encoding. We found that CNN with label encoding outperforms the other models but surprising; the testing accuracies are low. *K*-mer encoding is the best method for obtaining good testing and validation accuracy. This dataset cannot be evaluated only with accuracy metrics. Other metrics like precision, recall, sensitivity, and specificity also have to be considered. For a class with high samples, CNN with label encoding offers a high precision rate, and for a class with lower samples, CNN with *K*-mer encoding provides a higher precision rate. The recall value for all the models with *K*-mer encoding is high irrespective of class labels. If a high recall rate is preferred for a classification model, then *K*-mer encoding can be used. To obtain higher recall and sensitivity value for class with more sample, bidirectional LSTM with label encoding will be a good choice. CNN with label encoding offers a higher specificity rate for all the class irrespectively of class size. Thus, the encoding methods are selected based on the number of samples in the class and based on the required metrics to evaluate the model.

## Figures and Tables

**Figure 1:** DNA and RNA structure.

**Figure 2:** Distribution of each class and number of samples in a dataset.

**Figure 3:** Sample dataset with genomic sequences and their length.

**Figure 4:** Sequence data encoding using Label Binarizer.

**Figure 5:** Sequence data encoding using the *K*-mer technique.

**Figure 6:** Workflow of the proposed model for the classification of DNA sequence.

**Figure 7:** Architecture of the LSTM model.

The article "Analysis of DNA Sequence Classification Using CNN and Hybrid Models" was published in 2021. Journal: Comput Math Methods Med.

**Figure 8:** Architecture of bidirectional LSTM.

**Figure 9:** Confusion matrix of Label encoding and *K*-mer encoding for DNA sequence classification.

**Figure 10:** Accuracy of classification models.

**Figure 11:** Training and validation accuracy curve for Label and *K*-mer encoding.

**Figure 12:** Training and validation loss curve for Label and *K*-mer encoding.

**Figure 13:** Performance analysis of proposed method with various state-of-the-art methods.

**Table 1:** Metadata information of the dataset.

Column name	Type
Assembly	Number
SRA_Accession	Number
Release date	Date
Species	String
Genus	String
Family	String
Molecule type	String
Sequence	DNA sequence
Length	Number
Publications	Date
Geo_Location	String

**Table 2:** Complete architecture specification of proposed CNN model.

Layer (type)	Output shape	Param #
Embedding	(None, 1000, 8)	128
Conv1D_1	(None, 1000, 128)	3200
MaxPooling1D_1	(None, 500, 128)	0
Conv1D_2	(None, 500, 64)	24640
MaxPooling_2	(None, 250, 64)	0
Flatten	(None, 16)	0
Dense_1	(None, 128)	2176
Dense_2	(None, 64)	8256
Dense_3	(None, 6)	390

**Table 3:** Models performance concerning different class with Label and *K*-mer encoding.

Model class		Label encoding						*K*-mer encoding					
		a	b	c	d	e	f	a	b	c	d	e	f
CNN	Accuracy	0.93	0.99	0.92	0.99	0.99	0.99	0.93	0.99	0.93	0.99	0.99	0.99
	Precision	0.90	0.97	0.77	0.99	1.00	0.99	0.89	0.97	0.94	1.00	0.99	0.99
	F1	0.94	0.93	0.5	0.99	0.99	0.99	0.94	0.96	0.49	0.99	0.99	0.99
	Sensitivity	0.98	0.90	0.37	0.99	0.99	0.99	0.99	0.96	0.33	0.99	0.99	0.99
	Specificity	0.86	0.99	0.98	0.99	1.00	0.99	0.84	0.99	0.99	1.00	0.99	0.99

CNN-LSTM	Accuracy	0.93	0.99	0.92	0.99	1.00	0.99	0.93	0.99	0.93	0.99	0.99	0.99
	Precision	0.89	0.98	0.82	0.99	1.00	0.99	0.89	0.94	0.93	0.98	0.99	0.99
	F1	0.94	0.95	0.49	0.99	1.00	0.99	0.94	0.95	0.48	0.99	0.99	0.99
	Sensitivity	0.98	0.93	0.35	0.99	1.00	0.99	0.99	0.96	0.32	0.99	0.99	0.99
	Specificity	0.85	0.99	0.99	0.99	1.00	0.99	0.84	0.99	0.99	0.99	0.99	0.99

CNN-bidirectional LSTM	Accuracy	0.93	0.99	0.92	0.99	0.99	0.99	0.93	0.99	0.93	0.99	0.99	0.99
	Precision	0.89	0.95	0.84	0.93	0.98	0.99	0.89	0.98	0.94	0.99	0.99	0.99
	F1	0.94	0.82	0.40	0.96	0.99	0.99	0.94	0.96	0.48	0.99	0.99	0.99
	Sensitivity	0.99	0.72	0.26	0.99	0.99	0.99	0.99	0.95	0.33	0.99	0.99	0.99
	Specificity	0.84	0.99	0.99	0.99	0.99	0.99	0.84	0.99	0.99	0.99	0.99	0.99

## Data Availability

The data used to support the findings of this study are available at “The National Centre for Biotechnology Information (NCBI)” (https://www.ncbi.nlm.nih.gov).
